The article "Load Prediction Model of Athletes' Physical Training Competition Based on Nonlinear Algorithm Combined with Ultrasound" was retracted in 2023. Reasons: signs of a paper mill; suspected computer-generated content; unreliable results or conclusions; lack of ethics approval or compliance.

# Load Prediction Model of Athletes' Physical Training Competition Based on Nonlinear Algorithm Combined with Ultrasound

**DOI:** 10.1155/2022/3465556

**Published:** 2022-08-24

**Authors:** Zhiliang Zheng

**Affiliations:** Ulanqab Inner Mongolia Autonomous Region, Ulanqab Medical College, Wulanchabu City, Inner Mongolia 0474, China

## Abstract

In order to provide theoretical support and ideas for the “dose” of high-stakes physical activity in athletics, the author has developed models for athletic competition based on nonlinear techniques together with ultrasound. Based on test data, average mean estimation method, and nonlinear regression model estimates, 52 points (46 test points, 6 point estimates) is enrolled in the highest voltage and maximum voltage measurement based on the BP neural network model. The estimation method was developed and the accuracy of the estimation of our estimation method was compared and evaluated using the estimation data. Experimental results show that the average relative error of the average estimate compared to the accuracy of the bench press was 25%, the standard estimate which is not linear regression is 31%, and BP neural network model estimation is 9%. Compared with the accuracy of the assumption of half squatting, the average relative error of the estimated velocity is 13%, the standard nonlinear regression estimate is 20%, and BP neural network model estimated method is 9%. The BP neural network predicts the method with the best performance and intelligence, but its actual functioning and application are complex. The average speed estimate is the most appropriate for use, but the equipment must be high. The process of estimating a linear regression model requires minimal equipment, but its prediction error is high.

## 1. Introduction

Today, the competition in sports science and technology is increasing, and in order for sports to be successful, we need to have educational standards and procedures. Baking and athletics are competitions in science and technology. Achieving the concept that science and technology is a force to be reckoned with, implementing the concept of “competitive sports through science and education,” and improving governance and physical activity is a key element in the application of competitive science and technology in sports. Sports training and athletic science and technology are integrated [1]. Our research focuses on key issues in practice that meet the needs of real-world training, including social studies, public relations and more. Energy for the development of technology will support the extensive research of athletic training, fulfill the role of science research and technology, and improve the athletic skills of athletes.

The article "Load Prediction Model of Athletes' Physical Training Competition Based on Nonlinear Algorithm Combined with Ultrasound" was retracted in 2023. Reasons: signs of a paper mill; suspected computer-generated content; unreliable results or conclusions; lack of ethics approval or compliance.

The Chinese and their world-class rivals collect a lot of monitoring data during daily training and competition. Faced with these large amounts of data, how to comprehensively use it to help coaches and athletes improve their training levels and effects, achieve excellent results in competitions, and make these valuable data information play its due role is an urgent problem to be solved [2]. In response to this problem, the General Administration of Sports of the People's Republic of China put forward the requirement to develop a “national team information platform.” According to the different conditions of each national team, the informatization platform will be built in batches and in stages. In order to improve sports performance, it is necessary to carry out reasonable, systematic, and scientific training [3]. The importance of scientific training is to enable people to find the best way to maximize the potential of athletes, and the important premise of which is that athletes must have good physical function. The level of physical function directly affects sports quality and technical performance, which in turn affects sports performance. Therefore, it is necessary to regularly test and evaluate the physical function in each stage of training, and give feedback to the sports training, otherwise the training may not meet the training requirements or be terminated due to excessive fatigue.

## 2. Literature Review

In response to this research question, Zou et al. explored different data mining techniques for predicting match outcomes from the perspectives of football club managers and coaches, including decision trees, neural networks, Bayesian networks, and K-means algorithms, the experimental results show that the decision tree achieves the highest average accuracy in football match prediction [4]. Ethiraj and Dr performed data analysis of four consecutive football tournaments using random forest method to find the winning factors for winning the game [5]. Xue et al. simplified the scouting process of football players through data mining techniques and football industry standard data mining process methods, they developed and evaluated various classification models and regression models, the average accuracy for forward player positions in the classification model is 94%, and the minimum error for forward position in the regression model is 0.07, the results obtained through the model can simplify the work of scouts [6]. Bhargavi et al. used DEA and PageRank to rank college sports coaches, the ranking results can optimize coach allocation and game prediction, and provide decision support for allocating sports resources and personnel management [7]. Wang et al. proposed a new data mining method; to predict the outcome of college football games, they do not directly calculate the outcome of the game between two teams, but by looking for teams that are similar to their opponents, the prediction is made accoring to four aspects such as tactics and combat record [8]. Zhào et al. explored the application of association rules algorithm in badminton on-the-spot tactical analysis, used the improved association rules algorithm ACARMI to mine the game data, and found the tactical index that led to the loss of points [9]. Babai et al. discussed the application method of association rules and rough set theory in the field of tennis tactical decision-making, and combined with specific cases to find the main factors affecting the scoring rate of the game [10].

The article "Load Prediction Model of Athletes' Physical Training Competition Based on Nonlinear Algorithm Combined with Ultrasound" was retracted in 2023. Reasons: signs of a paper mill; suspected computer-generated content; unreliable results or conclusions; lack of ethics approval or compliance.

With the continuous development of modern sensing technology, it enables us to grasp the speed-force curve relationship in the process of strength training, and also lays a technical foundation for the successful implementation of optimal power load strength training. Many training benefits of optimal power load strength training are inseparable from the arrangement and monitoring of “dose load,” how to accurately determine the optimal power load is the primary factor in strength training practice [11]. Usually, determining the optimal power load requires a maximum strength test and an output power test. The process of testing the maximum strength is often time-consuming and labor-intensive, and athletes need to bear a certain risk of sports injuries. The process of testing the output power requires statistical analysis of the corresponding results obtained by the sensor equipment, and the coaches also need to arrange an appropriate training load to increase the accuracy of the test. In addition, the test process needs to be precisely controlled, and the requirements for the sensing equipment for collecting data, both greatly hinder the practical application of optimal power load strength training. In view of this, the author aims to solve the practical problem of determining the optimal power load, and constructs the average speed prediction method, nonlinear regression model prediction method, and BP neural network model prediction method of the optimal power load, and evaluates the accuracy of the three prediction methods. The “dosing” of high-level strength training load in competitive sports provides theoretical and practical support.  Figure 1 shows the load forecasting system based on nonlinear autoregressive neural network.

## 3. Research Methods

### 3.1. Research Objects

There are 52 male college students who are majoring in physical education at the University of Sports, 46 of them are experiments and 6 are estimates, all of whom have previous experience in weight training and strength training. All patients did not have multiple visceral disorders, liver and kidney function, and no abnormal behavior [12]. All courses have been informed in advance of the risks associated with participating in the experiment and signing a consent form. The main data of the topics are shown in Table 1.

The article "Load Prediction Model of Athletes' Physical Training Competition Based on Nonlinear Algorithm Combined with Ultrasound" was retracted in 2023. Reasons: signs of a paper mill; suspected computer-generated content; unreliable results or conclusions; lack of ethics approval or compliance.

### 3.2. Documentation Method

Using keywords such as “strength training”, “power”, “load”, “Strength Training”, “Power”, and “Optimal Power Load”, the relevant Chinese and English literature in CNKI, Wangfang Data, Google Scholar, Web of Science, PubMed, and other databases were searched, from the establishment of the database to March 30, 2020, 68 Chinese core journal papers and 2580 English journal papers were retrieved, including 8 Chinese and 112 English literature for key study, which comprehensively sort out the method to determine the optimal power load, and lay a solid theoretical foundation for this research.

### 3.3. Experimental Method

#### 3.3.1. Experimental Equipment

1 9-axis Bluetooth attitude sensor Wit-Motion (BWT901CL); 1 laptop; 2 sets of Smith racks (including standard barbell, barbell plate, fixed spring clip); 1 stopwatch; 1 roll of transparent tape; 1 external camera 1; and backup power supply 1.

#### 3.3.2. Experiment Process

(1) Determine the test indicators: according to expert advice and related research and experimental design, according to the principle that the movement structure in strength training is relatively simple, the technical impact is relatively small, the explosive force is mainly used, and the usability is the most extensive, the maximum strength of half squat and bench press as the load scheduling standard, and bench press throw and half squat as the evaluation index was determined. (2) Maximum strength test: using the NSCA test protocol, subjects were subjected to the bench press and semisquat 1RM test as the basis for the arrangement of strength training loads [13]. (3) Maximum output power test: strength training load is a continuous variable. The greater the test density, the stronger the fatigue of the subjects and the decrease of the test accuracy, according to the previous research design and pre-experimental test conditions, the maximum output power test of semisquat jumping and bench press throwing was determined under 10%, 30%, 50%, 70%, and 90% of 1RM load, and the load corresponding to the maximum output power is the optimal power load. Each level of load is required to collect valid data for one trial lift, and the interval time between groups is 2 to 5 minutes [14].

The article "Load Prediction Model of Athletes' Physical Training Competition Based on Nonlinear Algorithm Combined with Ultrasound" was retracted in 2023. Reasons: signs of a paper mill; suspected computer-generated content; unreliable results or conclusions; lack of ethics approval or compliance.

Before each test, subjects performed 15 min of regular warm-up activities, including 10 min of moderate-intensity jogging and 5 min of dynamic stretching, followed by a 3 min rest before the test. All strength tests are performed on a Smith stand with guards on both sides. In order to reduce the experimental test error: (1) Before the test, clearly inform the subject of the experimental action standard and organize the exercise; (2) Estimate its 1RM value according to the subject's height and weight; (3) Subjects were given verbal prompts and encouragements for each repetition; (4) No high-intensity resistance exercise was performed within 24 hours before the test; (5) The time interval between the maximum strength test and the maximum output power test was greater than 48 hours.

#### 3.3.3. Data Collection

MiniIMU (version number: 4.3.14) software is used to receive data, the transmission speed is 115200 bit/s, the recovery speed is 100 Hz, the speed is 0–8 gravitational acceleration, and the acceleration rate is offset, write the parameters, and select the time and acceleration of the output points. The special writing procedure is as follows: (1) Collect important information of the athletes. (2) The appropriate settings have been made in the software purchased by the operator to verify that the signal hardware is intact. (3) After setting up the test load, set the “prepare” password, and after the details appear on the Smith board, the operator will restart the software to zero. (4) When the training is completed, the test operator starts the purchase process in the computer recovery window, generates the instruction “3, 2, 1, start” password, and removes the contents from Smith's shelf and stores them after the test is complete. (5) Make a video of the complete collection of moving points [15].

#### 3.3.4. Data Processing

The output power, speed, and force value was calculated according to time, acceleration, and training load, the specific calculation formula is as follows

(1) $$\begin{array}{c} V_{i}=V_{i-1}+a_{i}\times t_{i},\\ F_{i}=m_{i}\times \left(a_{i}+g\right),\\ P_{i}=F_{i}\times V_{i}. \end{array}$$

Among them, *a* is the vertical acceleration, *V* is the instantaneous velocity, *P* is the output power, *m* is the training load, *g* is the acceleration of gravity (10 m/s^2^), and the initial velocity *V*_0_ = 0 m/s.

### 3.4. Mathematical Statistics

The data were summarized and calculated by EXCEL2007, and the obtained data were imported into SPSS22.0 for missing value, outlier and consistency test, one-way analysis of variance for significance test, and the GraphPad Prism Software 7.0 software for graph drawing [16]. All data are expressed by descriptive statistics such as mean (*M*), standard deviation (SD), among which the significant level is *P* < 0.05 and the very significant level is *P* < 0.01.

The article "Load Prediction Model of Athletes' Physical Training Competition Based on Nonlinear Algorithm Combined with Ultrasound" was retracted in 2023. Reasons: signs of a paper mill; suspected computer-generated content; unreliable results or conclusions; lack of ethics approval or compliance.

## 4. Results Analysis

### 4.1. Average Speed Prediction Method

Velocity-based training (VBT) refers to a training method in which the speed index of movement completion is used as the load standard in strength training. This method can arrange the strength training load according to the speed at which the movement is completed, estimate the maximum strength of the athlete, and monitor the training status of the athlete. In this part of the study, statistical analysis was carried out according to the different special experiences of the subjects. First, the subjects were tested with the maximum power output to determine the dynamic indicators at the maximum power output, and to lay a data foundation for the next analysis; secondly, the variance analysis was performed on the relevant indicators of the subjects at the maximum output power to verify which indicators had no significant difference between the various specialties and between the various mechanical indicators, and then to judge whether the speed prediction method was feasible; finally, the power-velocity curve relationship between semisquat and bench press tossing under different loads was established, and the average velocity value that can predict the best power load was determined.

### 4.2. Nonlinear Regression Model Prediction Method

A regression-dependent model is a form of function at more than one level at a different degree, and the law of regression is arranged on a graph based on the curves of various shapes, called nonlinear regression. A nonlinear regression model is a regression model with nonlinear models of unknown regression coefficients that generally represent nonlinear mathematical expressions between individual and nonlinear differences [17, 18]. The authors normalize power and training load, normalized power is the output power under different loads divided by maximum output power, and normalized training load is the relative load (training load/maximum strength). The bench press toss and the half squat were analyzed using nonlinear regression equations. The regression equation is specifically as follows:

(2) $$\begin{array}{c} \frac{P_{i}}{P_{\text{max}}}=b_{0}+b_{1}\left(\frac{L_{i}}{1\text{RM}}\right)+b_{2}{\left(\frac{L_{i}}{1\text{RM}}\right)}^{2}+b_{3}{\left(\frac{L_{i}}{1\text{RM}}\right)}^{3}. \end{array}$$

Among them, *P*_*i*_ represents the output power of different loads, *P*_max_ represents the maximum output power, *L*_*i*_ represents different training loads, 1RM represents the maximum strength, *b*_1_, *b*_2_, *b*_3_ represent regression coefficients, and *b*_0_ represents regression constants.

The article "Load Prediction Model of Athletes' Physical Training Competition Based on Nonlinear Algorithm Combined with Ultrasound" was retracted in 2023. Reasons: signs of a paper mill; suspected computer-generated content; unreliable results or conclusions; lack of ethics approval or compliance.

### 4.3. BP Neural Network Model Prediction Method

The author uses MATLAB2019b to establish a BP neural network model, adopts a three-layer topology, and takes the subject's height, weight, and maximum strength as the input layer, and the optimal power load as the output layer [19]. The number of neurons in the BP neural network model is determined by experience and trial and error, by comparing the network convergence speed and classification accuracy of the training set under the same conditions, it is finally determined that a reasonable number of hidden layer neurons in the prediction model is 10, the empirical formula for the number of hidden layer neurons is as follows:

(3) $$\begin{array}{c} M=\sqrt{N+L}+a. \end{array}$$

Among them, *M* is the number of neurons in the hidden layer, *N* is the number of nodes in the input layer, and *L* is the number of nodes in the output layer, *a* ∈ (1,  10).

Transformation of the BP neural network from the process into the latent layer is usually done using the tansig sigmoid tangent function as a function of the process latent neurons and normalizes the network release in the region area of [−1, 1]. The model estimates the sigmoid logarithmic function tansig based on the efficiency of the neurons in the output layer, changing the function from latent process to process output, linear function Pruelin, network operation function mse, number. The network iteration era is 1000 times and the learning speed is lr 0.05.

The experimental test data were input as training samples, and 70% of the total samples were randomly selected for the training set, 15% for the validation set, and 15% for the test set. They were calculated and modeled using the Levenberg–Marquardt algorithm [20].

As shown in Figure 2, after two times of learning, the BP neural network prediction model of the bench press tossed successfully converged, and the curve trends of the training set, validation set, and test set were generally consistent. The BP neural network prediction model was trained faster and had better training effect. Model fitting curve *R* = 0.77702, training set *R* = 0.72217, validation set *R* = 0.88723, and test set *R* = 0.86001, the data points are relatively evenly distributed near the fitting curve, the BP neural network model has good training effect, predictive power, and overall fit.

As shown in Figure 3, after 13 times of learning, the half-squatted BP neural network prediction model converges successfully, and the curve trends of the training set, validation set, and test set are generally consistent. The BP neural network prediction model has a faster training speed and good training effect [21]. Model fitting curve *R* = 0.82093, training set *R* = 0.87992, validation set *R* = 0.81067, and test set *R* = 0.85561, the data points are relatively evenly distributed near the fitting curve, the BP neural network model has good training effect, predictive power, and overall fit.

The article "Load Prediction Model of Athletes' Physical Training Competition Based on Nonlinear Algorithm Combined with Ultrasound" was retracted in 2023. Reasons: signs of a paper mill; suspected computer-generated content; unreliable results or conclusions; lack of ethics approval or compliance.

### 4.4. Comparison of Prediction Effects

The absolute error and the relative error are used as symbols to compare the accuracy of the estimates of our estimation method. The error is the difference between the estimated value and the measured value. The relative error is the percentage of the complete difference between the estimated value and the measured value in fact. The lower the value of the error and the relative error, the higher the accuracy of the estimation.

#### 4.4.1. Bench Press Toss Prediction Effect Comparison

The actual error is 6, the estimated value of the best load capacity of the new model chair press, and the average difference between the measured value, and the average relative. The approximate error is 6, the estimated value of the best energy. The estimated bench compression load is the same as the rated value 6, the lower the difference, the average percentage of the actual value, and the lower the relative force. It means that the higher the prediction accuracy is, the higher the prediction accuracy will be.

Comparing the requirements of the new model of 6 estimates, as shown in Figure 4, it can be seen that the inaccuracy of BP neural network hypothesis error is less than our estimate. The absolute value of the prediction errors of 4 forecasted objects is less than that of the nonlinear regression model prediction method, and the absolute value of the prediction errors of 6 forecasted objects in the nonlinear regression model prediction method is less than that of the average velocity prediction method [22]. The average error and the relative error of the BP neural network prediction method were 3.79 kg and 9%, respectively, of the average estimate of 8.50 kg and less than 25%, of which 9.33 kg and 31%, respectively, of the non-linear regression model estimation method. In general, the BP neural network prediction method is the best way to estimate the optimal strength of the estimation model, follow the average estimation method, and finally the nonhorizontal sample.

#### 4.4.2. Comparison of Prediction Effect of Half Squat

As shown in Figure 5, a hypothetical comparison of the new model of 6 estimates shows that the true rate of hypotensive error of the BP neural network is lower. Again in advance for our estimation procedures for estimating mean velocities and procedures for estimating nonhorizontal models. There are four ways to estimate the average velocity, and the accuracy of the estimated error of the estimated material is less than that of the nonhorizontal model [23]. The mean error and mean correlation error indicate that the error is incorrect and means that the relative error of BP neural network casino is 6.91 kg and 9%, fraction, which is less than 10.05 kg and 13% of the estimated velocity. For the method, it is less than 14.60 kg and is 20% of the estimated nonlinear regression model. In general, the BP neural network prediction method is the best way to estimate the optimal strength of the estimation model, follow the average broadcast estimation method, and finally the model nonlinear regression [24, 25].

The article "Load Prediction Model of Athletes' Physical Training Competition Based on Nonlinear Algorithm Combined with Ultrasound" was retracted in 2023. Reasons: signs of a paper mill; suspected computer-generated content; unreliable results or conclusions; lack of ethics approval or compliance.

## 5. Conclusion

The author has developed three approaches to estimating the optimal energy spectrum: the mean prediction rate, the standard nonlinear regression model, and the BP neural network prediction way. Among them, BP neural network predicts the possibility of having the best performance and intelligence, but its actual functioning and application are difficult. The average speed estimate is the most appropriate for use, but the equipment must be high. Nonlinear regression modeling techniques require less equipment, but the error prediction is larger and more appropriate for less trained athletes. It is suggested that when applying the optimal power load rapid prediction method for different strength training, it should be noted that the trial conditions should be on the Smith frame, and each trial lift should be completed with the same standard movements. When using free weight equipment for optimal power load strength training, the predicted value of the optimal power load can be adjusted appropriately.

## Figures and Tables

**Figure 1:** Load forecasting system based on nonlinear autoregressive neural network.

**Figure 2:** Training error curve of the optimal power load prediction model for bench press throwing.

**Figure 3:** Training error curve of the optimal power load prediction model for half squat.

**Figure 4:** Prediction results of optimal power load for bench press tossing.

**Figure 5:** Prediction results of optimal power load for half squat.

**Table 1:** List of subjects' basic conditions (*M* ± SD).

	Sample size	Age	Height/cm	Weight/kg	Bench press 1RM/kg	Half squat 1RM/kg
Testing object	46	22.11 ± 2.35	179.41 ± 3.31	72.21 ± 5.80	72.83 ± 15.97	124.93 ± 23.26
Prediction object	6	22.00 ± 1.79	177.50 ± 4.42	67.86 ± 4.29	66.67 ± 11.69	105.00 ± 22.58

The article "Load Prediction Model of Athletes' Physical Training Competition Based on Nonlinear Algorithm Combined with Ultrasound" was retracted in 2023. Reasons: signs of a paper mill; suspected computer-generated content; unreliable results or conclusions; lack of ethics approval or compliance.

## Data Availability

The data used to support the findings of this study are available from the author upon request.
